The article "Advanced Deep Learning Human Herpes Virus 6 (HHV-6) Molecular Detection in Understanding Human Infertility" was retracted in 2023. Reasons: unreliable results or conclusions; concerns about the data; concerns about the results or conclusions; concerns about the peer review.

# Advanced Deep Learning Human Herpes Virus 6 (HHV-6) Molecular Detection in Understanding Human Infertility

**DOI:** 10.1155/2022/1422963

**Published:** 2022-01-07

**Authors:** Malik Bader Alazzam, Ahmad Tawfig Al-Radaideh, Nasser Binsaif, Ahmed S. AlGhamdi, Md Adnan Rahman

**Affiliations:** ^1^Faculty of Computer Science and Informatics, Amman Arab University, Amman, Jordan; ^2^Department of MIS, College of Business, Jadara University, Irbid, Jordan; ^3^Department of E-Commerce, College of Administrative and Financial Sciences, Saudi Electronic University, Riyadh, Saudi Arabia; ^4^Department of Computer Engineering, Collage of Computers and Information Technology, Taif University, P.O. Box 11099, Taif 21944, Saudi Arabia; ^5^College of Business Administration (CBA), International University of Business Agriculture and Technology (IUBAT), Dhaka, Bangladesh

## Abstract

To see if HHV-6 may be a cause of infertility, researchers looked at 18 men and 10 women who had unexplained critical fertility and had at least one prior pregnancy. HHV-6 DNA was discovered in both infertile and fertile peripheral blood mononuclear cells (PBMC) (12 and 14%, respectively); endometrial epithelial cells from 4/10 (40%) infertile women were positive for HHV-6 DNA; this viral DNA was not found in the endometrium of fertile women. When endometrial epithelial cells were cultivated, they produced viral early and late proteins, suggesting the existence of an infectious virus. Endometrial HHV-6 infection creates an aberrant NK cell and cytokine profile, resulting in a uterine domain that is not favorable to conception, according to the findings. To corroborate the findings, studies of extra fertile and barren women should be done. Semen samples were taken from 18 guys who visited the Government General Hospital Guntur's infertility department because they were having reproductive issues with their partners. Herpes virus DNA has been discovered in the sperm of symptomatic fertile and infertile male patients on rare instances. Furthermore, researchers must investigate the role of viral diseases in male infertility.

## 1. Introduction

After a year of unprotected sexual intercourse, 15% to 20% of couples in European nations experience infertility. In roughly 33% of infertility cases, both male and female factors are present, up to 49.5 percent, depending on the fairness of the viral DNA detection technique utilized. Human herpes virus 6 (HHV-6) is a beta herpes virus with a strong link to human cytomegalovirus. Were the first to isolate HHV-6 from peripheral blood lymphocytes (PBL) obtained from lymphoproliferative clutter patients. Cell tropism is particularly notable for T lymphocytes, which was formerly dubbed human B-lymph tropic virus (HBLV). HHV-6A and HHV-6B are two hereditarily distinct strains of the virus. HHV-6 is a herpes virus that is related to HHV-7 and, to a lesser extent, human cytomegalovirus (HCMV). HHV-6 has been identified as a causative operator of exanthema subatomic (roseola), a common young exanthema, according to. HHV-6 illness is most common in the first two years of life. HHV-6 reactivates with immunological suppression, despite the fact that evident clinical illness is rare in adults. HHV-6 has been linked to a variety of human diseases, including multiple sclerosis (MS); however, the significance of these associations is unclear [1, 2]. The discovery of the HHV6 cell-surface receptor, as well as the confirmation of the hereditary groups of HHV-6A and-6B, is among the most recent discoveries in the subatomic science of HHV6. The discovery of the HHV-6 cell receptor, CD46, has provided yet another insight into HHV-6 cell tropism. In addition, the in vitro partnerships between HHV-6 and other viruses, particularly, the human immunodeficiency virus, and their significance for the in vivo situation, as well as the trans-activating limitations of a few HHV-6 proteins, are investigated. The clinical spectrum of HHV-6 is still being explored, and aside from being regarded as a significant pathogen among transplant recipients (as seen by the growing number of upcoming clinical tests), its role in focused sensory system disease is becoming increasingly obvious [3–5]. Finally, we offer a schematic depicting the many therapy options for HHV-6. The clinical spectrum of HHV-6 in immune-compromised people has occupied a large portion of the current literature on the virus. Reactivation of the beneficiary's strain, external illness in the contributor's strain, and reinfection with a different strain are all possibilities. In the bone marrow transplant population, a small number of individuals have been identified with interstitial pneumonitis caused by HHV-6, which is commonly associated with unit against host illness (GVHD) in the semen of asymptomatic infertile individuals [6].

The article "Advanced Deep Learning Human Herpes Virus 6 (HHV-6) Molecular Detection in Understanding Human Infertility" was retracted in 2023. Reasons: unreliable results or conclusions; concerns about the data; concerns about the results or conclusions; concerns about the peer review.

## 2. Materials and Methods

### 2.1. Clinical Samples

Eighteen males who went to the reproductive center at the GGH Guntur, Andhra Pradesh (from January 2017 to December 2017), owing to couple reproductive concerns, provided samples (1 ml) to verify the HHV-6 and twelve blood serum samples to test the antibodies to herpes virus. Every patient gave their informed permission for the purposes of the current examination. There were no clinical symptoms of HSV infection in the men who took part in the study, and no evident reasons of infertility were discovered. They were all sterile for unknown reasons. Individuals with any underlying disorders, such as diabetes, that might potentially interfere with fertility were excluded from the study.

Ten female patients were engaged for tubal patency testing and endometrial samples were collected from them [7–9]. The participants in the study had to be between the ages of 28 and 36 and have a normal menstrual cycle (20–32 days) and a BMI of 17.5 to 25.5 kg/m^2^. The menstrual cycles' secretory phase was planned (13 to 27 days). Tissue samples were obtained in HEPES-supplemented Dulbecco adjusted Eagle medium/Hams F-12 (DMEM/F-12).

### 2.2. Ethics Statement

A written consent was obtained from each patient, and ethics approval was obtained from the Ethical Committee of the medical centre.

All research studies involving human subjects necessitate the acquisition of research ethical approval. Before research subjects can be recruited or data collection can begin, this approval must be acquired.

### 2.3. Statistical Analysis

The data collected were analyzed with SPSS software version 15. The data were expressed as mean ± SD. The differences of variables between two groups HHV (+) ve versus HHV (−) ve were compared using the Student's *t*-test.

### 2.4. Analysis of Semen and Blood

A sperm count, commonly known as a semen analysis, determines the number and quality of a man's sperm and semen. The thick, white fluid discharged from a man's penis at his sexual climax is known as sperm (orgasm). Ejaculation is the term for this process. Sperm is the genetic material-carrying cell in a man's body. When a sperm cell combines with an egg from a woman, an embryo (the earliest stage of the development of an unborn baby) is formed.

Masturbation in sterile containers was used to gather sperm samples after 48–72 hours of sexual abstinence. Within 1 hour of collection, samples were evaluated, and within 2 hours of collection, samples were processed for DNA extraction. Computer-aided sperm analysis was used to analyze the sperm concentrations and motility of 18 male patients, according to the 4th edition of the WHO Guidelines. Observation of eosin-thiazine-stained methanol-fixed smears of fresh ejaculate under a light microscope and evaluation according to rigorous Krueger criteria were used to assess sperm morphology. Semen specimens that matched all of the aforementioned criteria were considered normal. The presence of an unusually large number of white blood cells did not indicate that the sample was abnormal. All sperm samples with one or more abnormal semen values were considered abnormal [10–14].

### 2.5. PCR Amplification Reactions and Extraction of DNA from Semen Samples

The molecular laboratory's core tools include DNA extraction and polymerase chain reaction (PCR). This brief overview covers the numerous physical and chemical procedures for extracting DNA in order to obtain adequate quantities of high-quality DNA. PCR can be used to increase the amount of DNA in a sample.

The article "Advanced Deep Learning Human Herpes Virus 6 (HHV-6) Molecular Detection in Understanding Human Infertility" was retracted in 2023. Reasons: unreliable results or conclusions; concerns about the data; concerns about the results or conclusions; concerns about the peer review.

To avoid contamination, all PCR test preparations were done in a “clean room” (no post-PCR DNA products) underneath a laminar flow hood. Each fresh semen sample was centrifuged for 30 minutes at 13,000 rpm after collection. The spermatozoa pellet was kept in the original Eppendorf tube, and the precipitate (seminal fluid) was transferred to a fresh one. In the event of a semen PCR test, sample DNA was collected using a DNA isolation from fluid Semen kit (QIAGEN; Cat no: 57704) according to the manufacturer's instructions. All participants' spermatogenesis and seminal fluids were tested for the presence of HHV-6 DNA using PCR with the appropriate set of primers (Table 1). Agarose gel in a 2 percent or 3 percent gel matrix, depending on the size of the PCR result, and then photography with an ultraviolet light transilluminator were used to examine the PCR results. Finally, to corroborate the initial amplification results, direct sequencing analysis of HHV 6 PCR products was done (Figure 1). The PCR products were purified using the QIAquick PCR purification Kit (Qian Valencia, CA) and then eluted with water [7]. DNA sequences were examined and identified by uploading them to the ribosome database project website [2].

## 3. Results and Discussion

### 3.1. HHV-6 in Women's Clinical Specimens

A whole blood quantitative PCR DNA test for HHV-6 is the most feasible way to find out if someone has chromosomally integrated HHV-6 (ciHHV-6). If the amount is greater than 500,000 copies per ml without an acute illness, the person has ciHHV-6.

In the current clinical study, ten women with unexplained primary infertility who had no past pregnancies or pathological variables were compared to 14 bigger women who had at least one previous successful pregnancy. Table 1 shows no significant differences between the two groups, save for a small increase in estradiol levels in infertile males (*P*=0.05; Student's *t*-test). Estradiol levels over a specific level may indicate that the hormone is suppressing the production of follicle-animating hormone (FSH) and that there are worries about richness. The amount of progesterone in the body did not change in any way.  Table 2 summarizes the outcomes of each clinical case based on whether or not HHV-6 infection was present. In one of the individuals' PBMCs, HHV-6 DNA was detected. Surprisingly, HHV-6 viral DNA was found in 44 percent of PCOS women's endometrial epithelial cells, but not in control women's cells (*P*=1.27 × 10 − 4; Fisher correct test). Similarly, no HHV-6 DNA and HHV-6A infection is restricted to the endometrial epithelium of primary infertile women, according to stromal cells recovered through epithelial cell purification (Table 2). Because HHV-6 dynamic illness is common in a group of infertile women, search for sharp disparities in markers, based on HHV-6 contamination (Tables 3 and 4). HHV-6 positive infertile women had greater estradiol levels than HHV-6 negative infertile women (*P*=0.045) (see Table 3, for further information.). Estradiol irregularities may have repercussions in HHV-6 infection, based on the discovery of a relationship. The proximity of HHV-6 infection was linked to estradiol dimensions (*P*=0.001; R2: 0.89; Spearman relationship). There were no clinical indicators that differed between the two spouses (Table 3). When we looked at immunological properties in the uterine state, we saw a shift in endometrial (e) NK cell-safe phenotype and cytokine levels. HHV-6 positive infertile women (8.06) had less CD56posCD16neg eNK cells than HHV-6 negative infertile women (23.82) (*P*=0.001) (for further information, see Table 4). CD56bright and CD56dim eNK cells were distributed differently in HHV-6A positive and negative infertile women, with HHV-6 positive infertile women (3.72) having less CD56bright and CD56dim eNK cells than HHV-6 negative childless women (13.68) (*P*=0.001) (for further information, see Table 4). Although there was no difference in the number of CD3+ lymphocytes between the two groups, there was a difference in the number of CD14+ monocytes (*P*=0.612). The uterine flushing aspects of cytokines presented an alternate example in both HHV-6 positive and negative infertile women [3–6].

The article "Advanced Deep Learning Human Herpes Virus 6 (HHV-6) Molecular Detection in Understanding Human Infertility" was retracted in 2023. Reasons: unreliable results or conclusions; concerns about the data; concerns about the results or conclusions; concerns about the peer review.

As a possible environmental cause of human infertility, viral infections have been connected. Although no single virus has been confirmed to induce female infertility, herpesviruses have been associated to male infertility in particular. In our study, furthermore, endometrial epithelial cells from infertile women exhibited high viral loads (about 4 copies of viral DNA per cell); no HHV-6A infection was found in stromal cells or PBMC, excluding the possibility of HHV-6 DNA being chromosomally integrated.

The frequency of the herpes virus in normal and abnormal sperm samples is shown in Table 4. According to the 4th edition WHO criteria, 9 of 18 sperm samples were classed as normal (normozoospermia). HHV6 viral DNA was found in 6 (33.3 percent) of normal sperm samples (Table 3). In 18 male individuals with aberrant zoospermia, viral DNA was also found (Table 5). The samples were further categorized into six oligozoospermic, five asthenozoospermic, three oligoasthenozoospermic, and four teratozoospermic subgroups in this group. In aberrant semen samples, HHV6 viral DNA was found in 4 (22.22 percent), 8 (44.44 percent), 2 (11.11 percent), 3 (16.67 percent), and 3 (16.67 percent) (Table 5). There was no significant statistical difference between the existence of each herpes virus and each aberrant grouping, according to statistical analysis. For at least one member of the herpes virus family, viral DNA was found by PCR in 16 (88.88 percent) of the 18 total semen samples (Table 5). The findings of viral DNA analysis for all 18 samples provided show that HHV-6 is present in 16 of them (88.88 percent). Previous research looked at the frequency of viral DNA in total sperm samples.

The mean sperm count and motility of virally infected and no infected semen samples are shown in Table 4. The mean sperm count after HHV-6 infection had no effect on mean sperm count. Kapranos et al. discovered that HHV1 infection was associated with decreased sperm count and motility. Previous research had revealed no link between HHV-6+ and HSV-6− DNA and poor sperm count, motility, or infertility.

### 3.2. The Difference between Normal and Abnormal Semen

Statistical analysis revealed no link between the presence of the herpes virus and the subsequent classification of samples as normal or abnormal semen, indicating that viral presence does not appear to have a significant impact on the semen's qualitative or quantitative features. Both normal and aberrant sperm had nearly identical amounts of viral DNA. HHV-6, on the contrary, appeared to be more common in oligozoospermic sperm than in asthenozoospermic sperm, although the difference was not statistically significant.

### 3.3. PCR Results and Gene Sequencing

In all three types of samples, including male and female, gel examination of PCR results revealed six bands in PCR amplicons for 2-globin gene fragmentation at 315 kb (Figure 1), with the appropriate primer sequence reported in Table 5. Figure 1 displays 7 bands of PCR amplification for U38 gene fragments on the right side, with positive control bands at 467 bp. Following the PCR form of HHV-6 virus isolates male (two kinds) and female samples, approximate sized DNA bands were produced. All viral isolates reacted well to the genes 2-globin (315 bp) and U38 (467 bp) among the two gene targets. In the current multi-PCR technology, 2-globin is moderately reflected.

## 4. Conclusion

Finally, for the first time, viral sickness caused by any of the seven herpes simplex viruses was discovered in both normal and pathological semen samples, suggesting that both groups had comparable high rates of viral illness. Herpes simplex is suspected of having a microorganism that affects sperm parameters and fertility. Overall, our data imply that HHV-6 infection in both men and women may lead to primary infertility.

The article "Advanced Deep Learning Human Herpes Virus 6 (HHV-6) Molecular Detection in Understanding Human Infertility" was retracted in 2023. Reasons: unreliable results or conclusions; concerns about the data; concerns about the results or conclusions; concerns about the peer review.

## Figures and Tables

**Figure 1:** PCR amplification for 2-globin gene (a) fragment (315 bp) and for U38 gene fragments (467 bp) (b).

**Table 1:** Demographic and clinical characteristics of women's cohorts (average values).

Parameters	Infertile (10)	Control (14)	*P* value ^*∗*^
Age (yrs)	33.4	33.8	0.93
Duration of infertility (yrs)	2.8	2.1	0.63
Length of menstrual cycle (days)	4.6	4.3	0.43
Follicle-stimulating hormone (FSH) (mUI/mL) (day 3)	9.1	7	0.41
Luteinizing hormone (LH) (mUI/mL) (day 3)	6.7	6.2	0.41
Estradiol (pg/mL) (day 3)	76.8	65.7	0.05
Thyroid-stimulating hormone (TSH) (uUI/mL)	2.4	1.9	0.44
Free thyroxine (FT4) (pg/mL)	1.8	1.1	0.85
Progesterone (pg/mL) (day 21)	11.67	13	0.53
Day (menstrual cycle) of sample collection	13.8	13	0.80

Student *t*-test.

**Table 2:** Infertile women were split into two groups based on whether or not they had HHV-6 infection: infertile and control women's demographic and clinical characteristics (average).

Parameters	HHV-6 positive	HHV-6 negative	*P* value ^*∗*^	Control (14)
Age (yrs)	33.4	32.8	0.84	33.8
Duration of infertility (yrs)	2.9	2.8	0.56	2.1
Menstrual cycle length (days)	4.8	4.6	0.38	4.3
FSH (mUI/mL) (day 3)	9.5	9.2	0.37	7.0
LH (mUI/mL) (day 3)	7.0	6.8	0.37	6.2
Estradiol (pg/mL) (day 3)	79.9	77.5	0.04	65.7
TSH (uUI/mL)	2.5	2.4	0.39	1.9
FT4 (pg/mL)	1.9	1.8	0.76	1.1
Progesterone (pg/mL) (day 21)	12.1	11.8	0.48	13.0
Day (menstrual cycle) of sample collection	13.2	12.8	0.72	13.0

Student *t*-test.

**Table 3:** Infertile women were split into two groups based on whether or not they had HHV-6 infection: endometrial samples immunological parameters.

Immune cells	HHV-6 positive	HHV-6 negative	*P* value ^*∗*^	Control
NK CD56posCD16neg (N)	8.06	23.82	0.001	24.78
NK CD56brightCD16neg (N)	3.72	13.68	0.001	14.89
NK CD56dimCD16− (N)	4.44	10.18	0.017	9.87
CD3+ (N)	0.00	0.00	0.000	0.00
CD14+ (N)	0.46	0.52	0.612	0.48

Student *t*-test.

**Table 4:** Mean sperm count and motility in virally infected and noninfected semen samples.

	Number of specimens	Sperm count (million/ml)	*P* value	Motility (mean)	*P* value
Viral DNA positive	9	27.67	0.71	38.53	0.67
Viral DNA negative	12	30.24	0.67	61.47	0.61
HHV-6 positive	16	29.67	0.91	70.14	0.5
HHV-6 negative	2	27.47	0.14	29.86	0.37

**Table 5:** Sequences of type-specific real-time PCR primers used for the detection of HHV6 in clinical samples.

Virus	Gene	Primers	Primer sequence (5′-3′)	Product size
HHV-6	*β*2-globin	Outer	GGA GAA GGT CTT′ CTC GGC CTC GTA GGC TTA GTA	315 bp
		Inner	GGT CGA GTC ATC TAC GGG GAC ACG GAA TTA GGC	

HHV-6	U38	Outer	ATT AAG TTG GTA GTA CTT ACG TGA TGG TTA GGA	467 bp
		Inner	GTA TTA GGA GGT TTG AAA GGT AAG TGA GGA GGT	

The article "Advanced Deep Learning Human Herpes Virus 6 (HHV-6) Molecular Detection in Understanding Human Infertility" was retracted in 2023. Reasons: unreliable results or conclusions; concerns about the data; concerns about the results or conclusions; concerns about the peer review.

## Data Availability

The data used to support the findings of this study are included within the article.

## References

[1] Dhanvijay M. M., Patil S. C. (2019). Internet of Things: a survey of enabling technologies in healthcare and its applications. *Computer Networks*.

[2] Domínguez-Mayo F. J., Escalona M., Mejías M. (2015). A strategic study about quality characteristics in e-health systems based on a systematic literature review. *The Scientific World Journal*.

[3] Eggert A., Ulaga W. (2011). Customer perceived value: a substitute for satisfaction in business markets?. *Journal of Business & Industrial Marketing*.

[4] Esmaeilzadeh P., Sambasivan M., Kumar N. The challenges and issues regarding e-health and health information technology trends in the healthcare sector.

[5] Fattah F. A. M. A., Mohamed A. H. H., Bashir M. I. A., Al Alawi A. M. M. (2020). Determinants of knowledge-sharing behaviour among students at higher educational institutions in Oman: a planned behaviour theoretical perspective of knowledge sharing. *Global Knowledge, Memory and Communication*.

[6] Häyrinen K., Saranto K., Nykänen P. (2018). Definition, structure, content, use and impacts of electronic health records: a review of the research literature. *International Journal of Medical Informatics*.

[7] Heo J., Han I. (2013). Performance measure of information systems (IS) in evolving computing environments: an empirical investigation. *Information & Management*.

[8] Hidayah N. A., Putri R. N., Musa K. F., Nihayah Z., Muin A. Analysis using the technology acceptance model (TAM) and DeLone & McLean information system (D&M IS) success model of AIS mobile user acceptance.

[9] Hsu J., Huang J., Kinsman J. (2015). Use of e-Health services between 1999 and 2002: a growing digital divide. *Journal of the American Medical Informatics Association*.

[10] Sengan S., Khalaf O. I., Priyadarsini S., Sharma D. K., Amarendra K., Hamad A. A. (2022). Smart healthcare security device on medical IoT using raspberry pi. *International Journal of Reliable and Quality E-Healthcare*.

[11] Sengan S., Khalaf O. I., Rao G. R. K., Sharma D. K., Amarendra K., Hamad A. A. (2022). Security-aware routing on wireless communication for E-health records monitoring using machine learning. *International Journal of Reliable and Quality E-Healthcare*.

[12] Zubair Z., aber R. (2021). A deep learning based optimization model for based computer interface of wheelchair directional control. *Tikrit Journal of Pure Science*.

The article "Advanced Deep Learning Human Herpes Virus 6 (HHV-6) Molecular Detection in Understanding Human Infertility" was retracted in 2023. Reasons: unreliable results or conclusions; concerns about the data; concerns about the results or conclusions; concerns about the peer review.

[13] Younis M. T., Al-kateeb Z. N. (2020). Application methods of linear feedback control on the modified lorenz 3D chaotic system. *Tikrit Journal of Pure Science*.

[14] Ali B. M., Younes B. (2013). The impact of information systems on user performance: an exploratory study. *Journal of Knowledge Management, Economics and Information Technology*.

